# Injury Related Risk Behaviour: A Health Belief Model-Based Study of Primary School Students in a Safe Community in Shanghai

**DOI:** 10.1371/journal.pone.0070563

**Published:** 2013-08-08

**Authors:** Ling-Ling Zhang, Koustuv Dalal, Shu-Mei Wang

**Affiliations:** 1 School of Public Health, “Key Laboratory of Public Health Safety, Ministry of Education”, Fudan University, Shanghai, China; 2 Centre for Injury Prevention and Safety Promotion (CIPSP), School of Health and Medical Sciences, Örebro University, Örebro, Sweden; University of Rochester, United States of America

## Abstract

**Aim:**

To explore the relationship between Health belief model (HBM) and children and adolescents' unintentional injury risk behavior, to add some useful information for injury prevention.

**Methodology:**

We investigated injury related health risk behavior and health belief status of students at primary schools grade 3 to 4, in a Safe Community, in Shanghai. Self-administered injury questionnaires were used to investigate risk behavior of students and HBM factors.

**Principal Findings:**

The prevalence of risk behavior among students reported in this community was high. HBM scores showed differences between two groups of students classified by whether they had risk behavior or not. Self-efficacy was highly related with the status of socio-psychological behavior.

**Significance:**

HBM has been widely used in explaining the disease-related behavior; however, it has been seldom used in injury-related behavior. The study demonstrated important relation of HBM to students' injury issues, and HBM could explain injury related behavior as well, especially for traffic injury-related behavior. When developing injury prevention strategies, we can take it into account.

## Introduction

Globally, injury is a major public health issue [1], [2]. Injury mainly occurs in younger population groups, especially among children and adolescents [1], [3]. Not only do injuries result in an increase in the number of deaths among adolescents than other causes, but also consume a majority of health care services [4], [5]. In China, of all the types of incidents that happen annually, nearly 200 million people are injured, often leading to fatalities of approximately 700,000 to 750,000 annually [6]. Since the 1990s, injury has replaced diseases as the leading killer among the primary and secondary school students in China [4], [5]. Injuries can cause disabilities, mental health disorders, and even deaths among young people [7], [8]. Moreover, injuries have inflicted huge economic loss and considerably impact families and society.

Recent studies are increasingly concerned about adolescent injuries and related risk behaviours [9]–[13]. Several academic theories are attempting to better explain the health risk behaviours. As a major conceptual framework for guiding the health behaviour change of individuals [14], the health belief model (HBM) has been widely used in explanation, prediction, and intervention of health-related actions in clinical practice [15], such as breast self-examination [16], [17]. Performance and utility of HBM has been fully confirmed through a large number of empirical studies [18]; however, scholarly application of HBM to adolescent unintentional injuries is limited [19].

In the Safe Community of Shanghai, major school programs are on health education and improvement of the campus environment. Each school has established a safety promotion project group. Diversified training activities have been carried out to disseminate safe community concepts, rules, and regulations on school and student safety. Each school has paid more attention to students' awareness of safety and started safety education courses. The current study investigated the injury related health risk behaviours and health belief status of primary school students in a safe community in Shanghai, China [20]. HBM has been used to explain risk behaviour, with the aim of providing relevant information for the development of unintentional injury prevention strategies for adolescents.

## Materials and Methods

### Participants

The study population was primary school students in a Shanghai community which had initiated the World Health Organization (WHO) Safe Community project in July 2009. There were seven primary schools altogether in the community. Five schools were randomly selected. Taking into account the characteristics of the cognitive development [21] and academic burden of students, we chose all of the 3rd and 4th grade students as subjects.

### Instrument and Procedure

We designed the self-administered questionnaire to investigate the health risk behaviours and health belief of the subjects. The questionnaire is mainly comprised of three parts: 1) injury related health risk behaviours, 2) health belief, and 3) self-efficacy. The reliability score of the whole questionnaire by Cronbach's alpha test was 0.947. The Cronbach's alpha for different parts of questionnaire mentioned above was 0.730, 0.958, and 0.829, respectively.

#### (1) Injury related health risk behaviours

Risk behaviour status of the students over the past 30 days was investigated. This section involved three major parts: 1) traffic injury related risk behaviours, 2) daily life injury related risk behaviours, and 3) adverse socio-psychological state. Of the total 18 questions, there were 5 items to assess traffic related risk behaviour (e.g., “I have crossed the road isolation rod or fence over the past 30 days”; “I have frolicked with others in the road”), 6 items for daily life injury related risk behaviour (e.g., “I do not warm up before sports”; “I play with knives, scissors, or other types of sharp tools”), and 7 items for adverse socio-psychological state (e.g., “I have been unfriendly teased”; “I have been in an unpleasant mood due to learning stress or academic performance”). Each item offered 3 response choices ranging from ‘frequently’ (scores 1 point), ‘occasionally’ (scores 2 points) to ‘never’ (scores 3 points). Participants rated their response to the items according to their actual situation. Furthermore, a lower score indicated more frequent risk behaviour. Score ranges are presented in table 1.

**Table 1:** Question distribution and question scores.

	N. of items	Score range	Cronbach's alpha
**Health risk behaviour**			
Traffic injury related risk behaviours	5	5–15	
Daily life injury related risk behaviours	6	6–18	
Adverse socio-psychological state	7	7–21	
**Dimensions of HBM**			
Perceived susceptibility	14	14–70	0.951
Perceived severity	8	8–40	0.862
Perceived benefits	6	6–30	0.897
Perceived barriers	4	4–20	0.836
Cues to action	4	4–20	0.855
Self-efficacy	10	10–40	0.829

#### (2) Health belief

According to HBM [15], it consists of the following dimensions: perceived susceptibility, perceived severity, perceived benefits, perceived barriers, and cues to action. The stronger the individual's health belief, the greater the likelihood of adopting healthy behaviour. In total 49 questions were designed based on HBM to assess each dimension. All items offered five response choices from “strongly disagree” (scores 1 point) to “strongly agree” (scores 5 points). Participants rated their response according to their actual situation. Score ranges are presented in table 1.

#### (3) Self-efficacy

We used the General Self-Efficacy Scale (GSES) [22] to assess whether subjects had confidence in controlling internal and external factors and succeeded in eventually adopting healthy behaviours. It consists of 10 items, all of which offered 4 response choices ranging from “completely incorrect” (scores 1 point) to “completely correct” (scores 4 points). A higher score indicates higher individual self-efficacy, which means that the student is more likely to adopt healthy behaviour.

### Ethical issue

Our study was approved by the Ethical Review Board of the School of Public Health, Fudan University. The study was a part of a large injury intervention program which was conducted among primary and secondary school students in Shanghai. Not only the students, but their parents and teachers were also included in the study. Self-designed questionnaires of good content validity and reliability on injury were used to gather related information. Parent questionnaires included a written consent form on the first page, in which the purpose and procedures were described in detail. Before the participation of the children, the parents needed to sign the informed consent. Following the written consent, we listed the parents and their children as subjects. The questionnaire survey was administered afterwards. However, if parents refused to participate, s/he and her/his child were excluded. In this paper, we only analysed the data extracted from the primary school student questionnaires, not the data involving parents or teachers.

### Data Analysis

In the primary analysis, we used the chi-square test and found significant statistical difference in the gender distribution of some injury related risk behaviours, meaning gender contributed to risk behaviours. Assuming that gender may serve as a covariate in the comparison of HBM dimensions, we carried out an analysis of covariance. After adjusting for the role of gender, we reported the mean difference and p value of each HBM dimension between groups. A database was established using Epidata version 3.1. All the data analysis was performed with SAS version 9.1.3 for windows. P<0.05 was considered statistically significant [23].

## Results

### Sample characteristics

In total, there were 948 students in the selected classes. In this study 932 questionnaires were eligible with the effective response rate of 98.3%. There were 513 boys (55.04%) and 419 girls (44.96%). Approximately 37.2% of the participants were grade 3 (n = 347), 62.3% were grade 4 (n = 585).

### Injury-related risk behaviour

The sample can be divided into two parts: students who had ever engaged in risk behaviours (occasionally/frequently) and students who had never engaged in risk behaviours. The distribution of students' risk behaviours is displayed in table 2. Generally, the percentage of students who had ever engaged in risk behaviours was low; however, it was relatively high in some specific behaviours, such as: “I do not warm up before the sports activities” (n = 421, 45.17%); “I do not use protective equipment in sport activities” (n = 352, 37.77%); “I have been unfriendly teased” (n = 447, 47.96%); and “I have been in an unpleasant mood due to learning stress or academic performance” (n = 564, 60.52%).

**Table 2:** The distribution of injury related risk behaviour (Number of students, percentage).

Category	Boy		Girl		Total			P
	Have ever engaged	Have never engaged	Have ever engaged	Have never engaged	Have ever engaged		Have never engaged	
**Traffic**								
1. I crossed the road isolation rod or fence over the past 30 days.	38	475	18	401	56	876		0.047
	7.40	92.60	4.29	95.71	6.01	93.99		
2. I ran the red light or did not take the zebra-crossing or the pedestrian over-pass or the underpass when crossing the road	121	392	88	331	209	723		0.347
	23.59	76.41	21.00	79.00	22.42	77.58		
3. I have frolicked with others in the street	45	468	26	393	71	861		0.142
	8.77	91.23	6.21	93.79	7.62	92.38		
4. I did not fasten my seat belt in a car or wear a helmet when I was on a moped/motorbike.	126	387	96	323	222	710		0.556
	24.56	75.44	22.91	77.09	23.82	76.18		
5. I rode on a vehicle (car or motorcycle) whose driver was drunk.	45	468	22	397	67	865		0.038
	8.77	91.23	5.25	94.75	7.19	92.81		
**Daily life**								
1. I did not warm up before sports activities.	236	277	185	234	421	511		0.572
	46.00	54.00	44.15	55.85	45.17	54.83		
2. I use protective equipment in sports.	323	190	257	162	580	352		0.610
	62.96	37.04	61.34	38.66	62.23	37.77		
3. I often play with matches, lighters or things like that.	77	436	29	390	106	826		0.001
	15.01	84.99	6.92	93.08	11.37	88.63		
4. I quarrel and fight noisily with others when eating or drinking water.	99	414	35	384	134	798		0.001
	19.30	80.70	8.35	91.65	14.38	85.62		
5. I played with knives, scissors, or other types of sharp tools.	87	426	76	343	163	769		0.637
	16.96	83.04	18.14	81.86	17.49	82.51		
6. I have provoked a cat, dog, or other pets.	159	354	145	274	304	628		0.242
	30.99	69.01	34.60	65.40	32.62	67.38		
**Adverse socio-psychological state**								
1. I have been unfriendly teased.	278	235	169	250	447	485		0.001
	54.19	45.81	40.33	59.67	47.96	52.04		
2. I have been asked for property and money.	56	457	26	393	82	850		0.012
	10.92	89.08	6.21	93.79	8.80	91.20		
3. I have been deliberately excluded by other students.	163	350	83	336	246	686		0.001
	31.77	68.23	19.81	90.19	26.39	73.61		
4. I have fought with others.	248	265	52	367	300	632		0.001
	48.34	51.66	12.41	87.59	32.19	67.81		
5. I have been in an unpleasant mood due to learning pressure or academic performance.	320	193	244	175	564	368		0.198
	62.38	37.62	58.23	41.77	60.52	39.48		
6. I have suffered from insomnia.	149	364	94	325	243	689		0.022
	29.04	70.96	22.43	77.57	26.07	73.93		
7. I have felt sad, hopeless, or depressed for more than 2 weeks.	89	424	48	371	137	795		0.011
	17.35	82.65	11.46	88.54	14.70	85.30		

For traffic injury related risk behaviours, proportions of girls (95.71%) who did not cross the road isolation rod or fence were higher than proportions of boys (92.60%). For daily life injury related risk behaviours, proportionally more boys played with matches or lighters (15.01%); quarrelled or fought during eating or drinking (19.30%) than girls (6.92% and 8.35% respectively). Proportionally more boys had been teased (54.19%), deliberately excluded by peers (31.77%); fought with others (48.34%); had insomnia (29.04%) and depression (17.35%) than girls (40.33%, 19.81%, 12.41%, 22.43% and 11.46% respectively).

### Comparison of HBM factors

The scores distribution of HBM factors and the comparison results between the two groups are separately displayed in table 3 (traffic injury related risk behaviours), table 4 (daily life injury related risk behaviours), and table 5 (adverse socio-psychological state). It is indicated in table 3 and table 5 that the average scores of HBM factors were significantly better in the group of students (both boys and girls) who had never engaged in risk behaviours than the other group. Overall, the boys had higher mean scores than the girls when we compared between ever vs. never. Significant differences of scores are displayed in each comparison of HBM factors in traffic injury related risk behaviours (table 3) except for the item of *cues to action* (lower score of *perceived barrier* was better). The only significantly differed score in adverse socio-psychological state was the item of *self-efficacy* (table 5). However, in daily life injury related risk behaviours (table 4), the group of students who had never engaged in risk behaviours had slightly lower scores than the other group in terms of average scores of every HBM factors although no significant differences were found.

**Table 3:** Comparison of HBM factors on traffic injury related risk behaviour.

Items	Have ever engaged		Have never engaged		Mean difference	p
	(n = 432)		(n = 495)			
	Mean of item score	S.D.	Mean of item score	S.D.		
**Perceived susceptibility**	3.71	0. 88	3.91	0.88	−0.205	0.000
Boys	3.62	0.95	3.96	0.87		
Girls	3.80	0.75	3.86	0.90		
**Perceived severity**	3.57	0.91	3.74	0.91	−0.162	0.007
Boys	3.55	0.92	3.78	0.89		
Girls	3.61	0.88	3.69	0.93		
**Perceived benefits**	3.88	0.99	4.14	0.89	0.269	0.000
Boys	3.83	1.00	4.18	0.87		
Girls	3.94	0.97	4.10	0.91		
**Perceived barriers**	2.50	1.09	2.31	1.18	0.200	0.008
Boys	2.16	1.13	3.00	1.42		
Girls	2.57	1.13	2.33	1.20		
**Cues to action**	3.40	1.05	3.47	1.09	−0.074	0.304
Boys	3.34	1.11	3.52	1.06		
Girls	3.46	0.96	3.41	1.12		
**Self-efficacy**	2.66	0.55	2.85	0.60	−0.189	0.000
Boys	2.68	0.60	2.85	0.60		
Girls	2.63	0.49	2.84	0.60		

SD  =  standard deviation.

**Table 4:** Comparison of HBM factors on daily life injury related risk behaviour.

Items	Have ever engaged		Have never engaged		Mean difference	p
	(n = 794)		(n = 123)			
	Mean of item Score	S.D.	Mean of item score	S.D.		
**Perceived susceptibility**	3.83	0.78	3.75	0.93	0.073	0.39
Boys	3.79	0.89	3.80	1.14		
Girls	3.86	0.79	3.72	1.04		
**Perceived severity**	3.66	0.87	3.64	1.12	0.019	0.833
Boys	3.66	0.87	3.72	1.17		
Girls	3.67	0.87	3.58	1.09		
**Perceived benefits**	4.02	0.92	3.99	1.06	0.03	0.740
Boys	4.00	0.94	4.06	1.08		
Girls	4.05	0.91	3.93	1.06		
**Perceived barriers**	2.37	1.11	2.55	1.33	−0.183	0.099
Boys	2.42	1.13	2.65	1.45		
Girls	2.31	1.08	2.45	1.23		
**Cues to action**	3.43	1.05	3.49	1.20	−0.051	0.628
Boys	3.41	1.08	3.64	1.17		
Girls	3.45	1.02	3.34	1.25		
**Self-efficacy**	2.76	0.57	2.75	0.70	0.018	0.759
Boys	2.76	0.59	2.86	0.75		
Girls	2.77	0.54	2.64	0.65		

SD  =  standard deviation.

**Table 5:** Comparison of HBM factors on adverse socio-psychological state.

Items	Have ever engaged		Have never engaged		Mean difference	p
	(n = 728)		(n = 189)			
	Mean of item score	S.D.	Mean of item score	S.D.		
**Perceived susceptibility**	3.79	0.79	3.91	0.85	−0.114	0.122
Boys	3.76	0.91	4.02	0.98		
Girls	3.83	0.80	3.84	0.95		
**Perceived severity**	3.64	0.89	3.75	0.99	−0.107	0.155
Boys	3.63	0.89	3.83	0.99		
Girls	3.65	0.88	3.69	0.98		
**Perceived benefits**	3.99	0.94	4.14	0.93	−0.148	0.058
Boys	3.96	0.97	4.28	0.81		
Girls	4.03	0.92	4.05	0.99		
**Perceived barriers**	2.40	1.10	2.38	1.31	0.012	0.899
Boys	2.43	1.13	2.56	1.38		
Girls	2.35	1.05	2.28	1.24		
**Cues to action**	3.41	1.06	3.52	1.12	−0.102	0.250
Boys	3.41	1.08	3.58	1.16		
Girls	3.42	1.04	3.47	1.10		
**Self-efficacy**	2.73	0.57	2.86	0.64	−0.130	0.007
Boys	2.75	0.60	2.91	0.65		
Girls	2.72	0.52	2.83	0.64		

SD  =  standard deviation.

## Discussion

This study reveals that the reported prevalence of primary school students' injury related-risk behaviours in this community were not positive. The percentage of students in general who had ever jaywalked was 22.42% and who do not use seat belts/helmets when riding vehicles was 23.82%. The percentage of red light violators was higher than the national figure (12.2%) reported by the study on health risk behaviours of Chinese adolescents [24]. Before physical activities, appropriate warm-up stretching and use of protective equipment (e.g., knee pads, helmet) are necessary in reducing the risk of sport-related injury [25], however, our findings show that the percentages of students who do not warm-up or use protective equipment was as high as 45.17% and 37.77%, respectively. The serious consequence of unintentional injury [25], [26] is a great cause of concern, which calls into attention the need to regulate driving and sports behaviours of students.

In general boys were more exposed to injury related risk behaviour than girls. This is supporting previous findings [20]–[22], [24], [26]. Meanwhile, 47.96% of students reported that they had been unfriendly teased at least once in our study. The number was so large that it deserves serious attention. Bullying among youngsters is common in industrialized countries and has severely threatened youth development [27]. The aggressive behaviour may be verbal, physical, or psychological. Bullying should not be simply considered as a normative aspect of youth development. Not only does it have a strong association with serious campus violence such as weapon-carrying, and fighting-related injuries [28], but also may involve more aggressive behaviours and even suicide [29], causing the victims and the bullies to suffer long-term social, physical, and psychological harm [30]. Bullying at school must be addressed with due priority and further studies on intervention are warranted. We have also found that the adverse psychological status among students is prevalent; especially the percentage of pupils who “have been in an unpleasant mood due to learning stress or academic performance” is 60.52%. The figure is much higher than that of previous findings in 2005 (24.8%) [26]. In recent decades, since the introduction of competitive educational programs, academic performance has been highly valued. The increasing academic burden and unpleasant study environment have produced mental and psychological stress in students as revealed by several studies both in China and abroad [29], [31]. Negative mental state due to stressful life events and school work problems are responsible for adolescents' violence, alcoholism, drug addiction, and even suicide [32]. However, the state of mental healthcare has not been sufficiently addressed in many developing countries [33]. Based on the epidemic of adverse mental state manifested in the study, relevant psychological interventions are urgently needed for the promotion of mental health.

The health belief model has traditionally been used for the explanation and prediction of the individual behaviours [34]. In our study, we applied the constructs of HBM to explain the three types of dangerous behaviours and found that there were significant differences in almost all scores of HBM factors of traffic behaviours between the two groups. However, significant differences were only detected in *self-efficacy* in the adverse socio-psychological state. We can conclude through comparison that the health belief model exhibited better application in explaining the former type of risk behaviours, while slightly satisfactory for the latter. There may be several reasons to explain these findings. First, the former type of risk behaviours usually causes more visible injuries such as physical injuries, disabilities, and even death. Second, because of the adverse impact of economic fluctuation and limited resources, the investment priority of health resources has always been assigned to visible physical injuries or diseases. Mental health care has never received due attention. Concerning the close relationship between HBM factors and individual health risk behaviours, we can integrate mental health into general health education and promotion and put forward corresponding injury prevention strategies in the future. When formulating traffic injury prevention strategies, we should consider *perceived susceptibility, perceived severity, perceived benefits,* and *perceived barriers*; as for psychological intervention, we should focus on *self-efficacy*. We should support young people, help them rebuild their confidence, improve self-efficacy, and deal with life stress events in a positive way.

A limitation of the study is that all the data was self-reported. In the questionnaires, the students were required to recollect what had happened over the past 30 days thus recall bias and reliability can be problems, especially when the questions they were asked involved disobeying rules (e.g., traffic rules) or sensitive issues (e.g., being bullied or suffering from insomnia). Also, in the questionnaire we did not give concrete definitions to evaluate the frequency of the risky behaviours such as *frequently, occasionally,* and we realize that everyone has their own definition of *frequently, occasionally.* This inevitably impacted the results, which drew our attention to the necessity of more precise questionnaire design in the future. In addition, the source of the sample was relatively concentrated, as the subjects were all from the same safe community thus the extrapolation of the findings are limited. Consequently, one can define our research as a pilot study, and findings and experiences can be utilized in future studies in regional and national settings. Therefore, the results of this study should be considered taking into account these limitations.

## Conclusion

This study reveals that although apparent progress has been achieved in health education and promotion at primary schools in recent years, the need for improvement still exists. Further research and more effort are needed, especially on how to make the best of HBM theory to conduct intervention strategies of unintentional and intentional injuries on campus and establish comprehensive health-promoting schools.
